The article "The Application of Focused Care Model in the Management of Hepatitis B Patients in a Tertiary Care Hospital and the Impact on Patients' Quality of Life" was retracted in 2023. Reasons: unreliable results or conclusions; lack of ethics approval or compliance; concerns about the data; concerns about the peer review.

# The Application of Focused Care Model in the Management of Hepatitis B Patients in a Tertiary Care Hospital and the Impact on Patients' Quality of Life

**DOI:** 10.1155/2022/7770955

**Published:** 2022-09-12

**Authors:** Jian-Wei Zhang, Yan Wang, Hai-Hong Shan, Jia-Yu Duan, Juan Yu

**Affiliations:** ^1^Department of Infection, Shanxi Norman Bethune Hospital, Taiyuan, Shanxi Province 030000, China; ^2^Preventive and Health Care Department, Shanxi Norman Bethune Hospital, Taiyuan, Shanxi Province 030000, China

## Abstract

Chronic hepatitis B is one of the common infectious diseases in the world, with a wide epidemic range and strong contagiousness, which is difficult to completely eradicate. From July 2020 to April 2022, 142 patients with hepatitis B who were admitted to tertiary hospitals were selected and randomly divided into 2 cases, with 71 cases per case. The control group adopts a conventional model, and the observation group implements a nursing model based on the control group. The management capacity and quality of life before and after the two groups of care were compared. 94 patients with chronic hepatitis B who were admitted to the hospital from July 2020 to April 2022 were selected, and 47 cases were divided into the control group and observation group according to the admission time. The control group is given a conventional model, and the observation group is given a nursing model on the basis of the control group. Both groups of patients observed anxiety self-assessment scale (SAS), depression self-assessment scale (SDS), short life span scale (SF-36) scores, and treatment conditions before and after the intervention, to explore the application of nursing model in the management of hepatitis B patients in tertiary hospitals and its impact on patient quality of life. Based on study's precare outcomes, there was no statistically significant difference between the self-administered scale (PIH) score and the quality of life measurement summary scale (QOL-BREF) score (*P* > 0.05) between the two groups. After one month of care, both groups had lower PIH scores than before care, and QOL-BREF scores were higher than before care (*P* < 0.05). After one month of treatment, the PIH score of the observation group was significantly reduced, and the QOL-BREF score after one month of treatment was significantly higher than that of the control group (*P* < 0.05). The SAS and SDS scores in the observation group were lower than those in the control group, and the quality of life scores and treatment compliance were higher than those in the control group, and the difference was statistically significant (*P* < 0.05). *Conclusions*. The nursing model can effectively improve the management and quality of life of hepatitis B patients. It also had a significant positive effect on the therapeutic capacity and quality of life of patients with hepatitis B and improved patient compliance behavior and quality of life.

## 1. Introduction

Chronic hepatitis is one of the most common infectious diseases in the world, with wide coverage and strong infectivity, which cannot be completely cured. According to incomplete statistics, at this stage, the world's 2.4 pieces of Wuhan city is about 100 million day and night feeling hepatitis virus infection, about 686,000 people die day and night every year in Wuhan, and there are about 93 million hepatitis carriers across the country. Hepatitis is a contagious disease caused by viral infection. If the treatment fails, it is likely to develop cirrhosis of the liver ascites or advanced liver cancer, which is a great threat to the patient's life. There is no reasonable treatment for this disease, and patients must take long-term medication to alleviate the disease [1].

In the process of clinical treatment, patients do not have enough grasp of the disease, have poor management methods, and have behaviors such as self-return and drug discontinuation, resulting in ineffective disease control [2]. Relevant studies have found that better health services are conducive to improving patients' long-term self-control ability, improving clinical manifestations, alleviating disease, and improving the quality of daily life. Therefore, it is important to give the patient the necessary nursing intervention when treating the patient. At the same time, in the treatment of unrelated seriously harmful diseases in patients with hepatitis, efficient nursing interventions play a vital role in the efficacy and quality of life of patients. On this basis, this study selected 142 patients with hepatitis in tertiary hospitals to discuss the impact of care on the management level and quality of life of patients with hepatitis, and the conclusions are reported as follows [3].

The article is dedicated to discussing the impact of nursing style on the management level and quality of life of patients with hepatitis and has important research significance for the efficacy and quality of life of patients with hepatitis.

## 2. State-of-the-Art Technology

### 2.1. The Need for Health Education on Chronic Hepatitis B

Health education knowledge is also a programmatic, organized, and comprehensive science education theme activity, so that people are aware of healthy individual behaviors and lifestyles, prevent diseases, and promote the quality of health and life. At the same time, health education knowledge is conducive to patients to establish the confidence to correctly understand the disease and defeat the disease, so that patients can grasp the health care and medical expertise, closely cooperate with the treatment, and obtain medical results. The research of many scholars around the world has found that diffuse hepatitis is a typical physical and mental disease, which integrates physical diseases and psychological and social factors “three-dimensional.” Prolonged negative psychological conditions can also cause diseases of the central nervous system and reduce liver volume. However, many patients with diffuse hepatitis have little understanding of life and life path. Rest and regression of exercise, dietary structure, pharmaceutical knowledge, and disease are at different stages [4]. Further reduction of the patient's immune function is not conducive to the elimination of the human body, aggravating the disease and producing a variety of negative effects, forming a vicious circle, resulting in the onset of the disease [5]. Guo Jinlong et al. investigated the level of professional knowledge of hepatitis prevention in healthy populations and found that the basic knowledge level of hepatitis prevention in healthy populations accounted for 89%, and the illiterate group only reached 11%. Through investigation and analysis, Zheng Jie et al. found that such patients understand the causes of hepatitis, medication knowledge, life care, and how to exercise, disinfect and sterilize, and protect [6].

The professional knowledge participation rate of patients with hepatitis in our country is low, usually in backward areas, because our level is low, and the level of patients in large urban areas is high. However, due to busy work and no time to take care of it, Wuhan city seriously lacks health education knowledge about hepatitis, and the cognition of this disease is still stuck in a low level. Abnormal physiological effects, unhealthy habits, dietary mix and lifestyle, and other healing factors are ignored, causing hepatitis attacks [7]. For example, Chen Haiyan found in “Influencing Factors of Creating Healthy Behaviors and Preventive Measures for Secondary Hospitalization of Patients with Diffuse Hepatitis” that the second hospitalized patient had bad habits, living habits, and poor mentality [8]. Depending on the individual behavior of creating a healthy lifestyle for these patients, radical adherence to treatment may reduce seizures or reduce seizure levels [9]. Therefore, the implementation of dependent health education for patients with acute and chronic hepatitis and medical staff can reduce the level of healthy China and have important practical significance for reducing medical expenses and health expenditures of the broad masses of the people. This is shown in Figure 1.

### 2.2. Research Progress on Adherence and Its Influencing Factors in Patients with Chronic Hepatitis B

Patient compliance is defined as “the level at which the patient's behavior in the changes in medications, dietary combinations, and lifestyle habits is consistent with the doctor's order.” The word “listen” was first used by Chinese experts from Ruan to teach Chinese translation applications [10]. The emphasis on adherence refers to the level at which the patient's actions are consistent with the scripting written by the doctor in advance in the treatment and prevention of the disease. Because the disease of diffuse hepatitis is very long and prone to onset, many patients have little understanding of the condition and cannot carry out outpatient follow-up visits, take medicines, and change bad eating habits and living habits according to the medical instructions of medical staff. It can be seen that the efficacy of patients with hepatitis disorders is not ideal, and it is related to the cause of the disease; in addition to the lack of efficient therapeutic drugs, a key that cannot be ignored is the poor compliance of patients [11].

Obstacles to patient compliance are numerous and complex, including patients, physicians, medical security systems, and regulatory factors that affect each other. Patient compliance depends entirely on the patient himself, and promoting patient compliance must be coordinated by patients, physicians, medical treatment, etc. and can only rely on the efforts of patients. Some experts and scholars have summarized the key obstacles that may cause a decline in compliance. It can be solved from three different levels, doctor and patient, patient and medical, and doctor and medical treatment, and promote patient compliance. At this stage, the scientific research on factors that harm patient compliance is mainly in many aspects such as high blood pressure, diabetic patients, schizophrenia, epilepsy, tuberculosis, and “kidney transplantation” [12]. When analyzing the factors that endanger the treatment compliance of patients with chronic diseases, it is emphasized that the sociodemographic economic characteristics of patients are related to treatment compliance, including the elderly, disease characteristics, surrounding environmental applicability, doctor-patient contradictions, cognitive ability of treatment and disease, and beliefs in physical and mental health [13]. Literature data show that the current stage of treatment compliance in patients with hepatitis disorders is relatively scattered, and there is a lack of comprehensive assessment of adherence to patients with hepatitis diseases and the analysis of harmful compliance factors. Factors related to compliance have been found only in certain references. Drug use, patient perceptions of the importance and effectiveness of drugs, perceptions of the disease, concerns about adverse drug reactions, and doctor-patient conflicts may affect patients' self-adjusting personal behavior [14]. The details are shown in Figure 2.

### 2.3. Efficacy of Health Education on Chronic Hepatitis B

With the change of modern medical models from medicine to social medicine, doctors and nurses slowly realized that diffuse hepatitis is a typical physical and mental disease. Integrating the influencing factors of physiological diseases, psychological state, and social development, patients with diffuse hepatitis are not only physically uncomfortable but also bear various pressures in work, life, and thought, coupled with the lack of disease awareness and health care medical knowledge, repeated attacks of diseases, and long-term acceptance of therapeutic health education which has become a way for contemporary medical staff to recognize patients' diseases and health knowledge and their effectiveness [15]. This is to let people shape the concept of “better than cure,” develop good living habits, correct bad habits that are harmful to health, then maintain physical health, reduce the occurrence of diseases, or maintain physical health, and reduce the production of diseases or auxiliary treatment methods for curing diseases. Specifically guide hospitalized patients to read articles health education guidelines, and carry out systematic software health education according to their specific guidance, group special lectures, etc. [16]. The results show that health education is conducive to patients' learning knowledge and self-management ability, completing the long-term unification of professional knowledge, information content, and personal behavior in their physical and mental health. Gulalai et al. [17] carried out all-round education for hospitalized patients, so that patients could grasp the triggering elements of recurrence, grasp their own nursing knowledge, reduce the recurrence rate, and reduce the quality of life [18]. Satisfactory practical results were obtained. Through some forms of health education theme activities, patients have a better understanding of the treatment and health knowledge of acute and chronic hepatitis, and the poor living habits are greatly improved. According to health education, patients with diffuse hepatitis are made aware of the importance of medical treatment and antiviral treatment of nucleoside (acid) analogues in the infectious disease department or hepatology department of the hospital on time after the onset of the disease, especially according to health education, under the premise of timely, biochemical, excessive examination to prevent lesions, early detection of diseases, and timely treatment.

Therefore, health education for patients with diffuse hepatitis is used to grasp the factors that influence relapse, thus repairing patients' perception of life care and self-confidence in overcoming difficulties, so that they can move from passive therapeutic care to active prevention of disease and relapse [19].

### 2.4. Current Status of Health Education for Chronic Hepatitis B

In the past, under the influence of modern medical models and Western countries, China's health education has shown higher professional knowledge and technicality, but it does not attach great importance to service. With the change of scientific research on the meaning of physical and mental health in various countries in the world, medical personnel around the world have gradually begun to attach great importance to health education and will no longer regard it as a service but will closely integrate professional knowledge, technology, and services, that is, the quality and level of services to meet the needs of patients. Health education is rooted in our country, and Western theories and methods cannot be applied in a simple and mechanical way. It is necessary to combine the personality characteristics, mentality, and day and night physiological state of the Chinese nation in Wuhan City, China, and make full use of many unique health education methods created by Chinese medicine in the development of Chinese culture in the past five thousand years [20]. TCM hospital shoulders the daily task of applying TCM to prevent and treat diseases, ensure people's health, provide TCM health care services for the people, and inherit and develop academic research talents in TCM. However, under the situation of fierce competition in the diagnosis and treatment market, the diagnosis and treatment services of Chinese medicine hospitals are significantly lower, and it is impossible to maintain survival and development. Specific performances are as follows: first, in the introduction of many outstanding talents in Western medicine, the staff of traditional Chinese medicine is gradually reduced. Second, because of the low cost of traditional Chinese medicine services, it is expected to introduce many large- and medium-sized testing instruments to increase profits and maintain the rapid development of hospitals by carrying out surgeries and treatments in Western medicine. For a long time, China's hospitals have not had the characteristics of traditional Chinese medicine, and health education has no characteristics. The health education of patients with diffuse hepatitis in China must be closely integrated with the basic theories of traditional Chinese medicine such as “identity verification,” “future treatment,” and “four seasons of health care.” The health education of patients with chronic hepatitis should be closely related to the basic theories of traditional Chinese medicine such as “physical fitness identification,” “treatment,” and “four-hour diagnosis and treatment” and make full use of the characteristics of traditional Chinese medicine to create health education with the characteristics of traditional Chinese medicine. Health education has become one of the disciplines of great concern to the nursing profession at this stage. Its essence is an intervention, to give people the professional knowledge, technology, and services needed to change their personal behavior and lifestyle, so that when faced with health problems such as health and disease prevention, treatment, and recovery, they can carry out personal behavior selection, remove or reduce the sources of risk affecting health, and actively adopt healthy personal behaviors and lifestyles. In general, the medical care of patients with hepatitis is not only related to hospital equipment, medical water equality, and objective reasons. It is also related to the interference of objective factors such as the psychological state of nursing staff and personal behavior. The high emphasis on nursing models and the subjective interference of medical staff in the daily life of questioning hepatitis patients is reasonable, and the relationship between the factors is shown in Figure 3.

## 3. Investigative Methodology

### 3.1. Data Collection

142 patients with hepatitis B admitted to the hospital from July 2020 to April 2022 were studied. Selection criteria are as follows: (A) inclusion criteria: (1) CHB confirmed by serology, quantitative hepatitis B virus, and liver function; (2) have clinical symptoms such as liver discomfort, fatigue, and loss of appetite; (3) no cognitive impairment; and (4) acute medical history and (B) elimination criteria: (1) end-stage liver disease; (2) accompanied by other chronic diseases; and (3) those who do not have basic communication skills and cannot cooperate with the investigation. Enrolled patients were randomly divided into two groups of 71 cases each. In the observation group, there were 36 males and 35 females. The age ranges from 20 to 63 years, with an average of 38.62 ± 5.31 years. In the control group, there were 35 males and 36 females. The age ranges from 21 to 64 years, with an average of 38.34 ± 6.48 years. Comparing the general data of the two groups, the difference was not statistically significant (*P* > 0.05) and was comparable.

94 patients with hepatitis B admitted to the hospital from July 2020 to April 2022 were selected, all diagnosed by HBV-DNA ultrasound and laboratory-related tests, and the >2000 U/ml exclusion criteria are as follows: (1) combined malignant tumors and severe cardiopulmonary insufficiency, (2) hypersensitivity to the drug under study, (3) abnormal mental or consciousness, and (4) during pregnancy and lactation. The patients were divided into a control group and an observation group according to the admission time, with 47 cases each. In the control group, there were 26 males and 21 females The age ranges from 24 to 78 years, with an average of 57.6 ± 9.2 years. The course of the disease varies from 1 to 8 years, with an average of 4.4 ± 1.3 years. There were 24 males and 23 females in the observation group. Age ranges from 23 to 75 years, with an average of 55.6 ± 8.5 years. Lesions are 1 to 7 years, with an average of 4.3 ± 1.2 years. Clinical data were similar in terms of sex, age, and course of the disease in both groups, as shown in Figure 4.

### 3.2. Methods of Care

The control group adopted a conventional model, including issuing a health promotion manual, explaining hepatitis B-related knowledge in detail, conducting psychological guidance, and guiding patients to take drugs regularly and quantitatively.

The observation group implemented the nursing model on the basis of the control group, where there are two measures: cognitive interventions and behavioral interventions. Care options include the following: (1) psychological nursing: responsible nurses enable patients to express unhappiness in their hearts through verbal communication and achieve effective release of emotions. For patients with more serious psychological problems, one-on-one psychological counseling is given, and at the same time, when the patient is in a bad mood, use relaxed and pleasant music to channel bad emotions. Family members are encouraged to give psychological support to patients so that they can be psychologically comforted. (2) Cognitive health care: introduce patients to the pathogenesis, disease regression, clinical manifestations, transmission routes, and treatment measures of hepatitis B with easy-to-understand illustrations and language, disseminate relevant disease information, combine cases and good treatment effects, and establish patient cognitive therapy. (3) Behavioral health care: it is recommended that patients choose low-fat and high-protein foods such as eggs, lean meat, and fish, eat more fruits and vegetables, and increase vitamin supplements. Eat regularly, eat lightly, eat less, avoid spicy and other irritating foods, overeat, smoke and drink alcohol, and ensure adequate sleep. Patients are encouraged to perform moderate aerobic exercise (e.g., walking and tai chi) for 30 to 50 minutes each time. (4) Out-of-hospital nursing: publish the contact information of the attending physician when discharged, guide the patient to take the medication on time and review it regularly and seek medical treatment in time under special circumstances to prevent treatment delays. Establish WeChat and QQ groups, check messages regularly every day, and answer questions from patients and their families. And timely release of the latest news related to the disease.

The two measures of cognitive and behavioral intervention are as follows: (A) cognitive intervention. Based on the results of the patient's cognitive assessment, a targeted cognitive intervention plan was developed for them. (1) Comprehensive health education: use one-on-one communication to let patients understand the causal relationship and precautions of hepatitis B. Inform the patient in detail of the stage of the current treatment goal and the benefits of actively cooperating with the care, and fully improve the patient's confidence. Strengthen the health knowledge education of patients' family lies and improve their awareness of hepatitis B, so that they can fully give patients emotional care and actively cooperate with relevant care. (2) Conduct regular missionary lectures: distribute self-made hepatitis B publicity materials, including modules such as basic knowledge of diseases, life care, and rehabilitation exercises. At the same time, the missionary atmosphere is actively carried out, collecting each patient's questions, interacting with patients through scenario reenactment, and allowing nursing staff to record the minutes of each missionary meeting, summarize and organize them into leaflets, and send them to patients after the meeting to deepen their understanding and memory. (B) Behavioural intervention: (1) diet structure: develop a reasonable diet plan for patients, eat less and more meals, containing high protein and vitamins, etc., a balanced diet, and recommend that patients quit smoking and alcohol. (2) Exercise and rest: bed rest is the main focus of patients during acute exacerbations, avoid unnecessary activities, and ensure adequate sleep. (3) Drug intervention: during hospitalization, by quoting the opposite word, patients are instructed and advised to take the drug regularly and quantitatively and are told to stop the drug without authorization or reduce the harm caused by the use of the drug. After discharge, a love contact card is issued to each patient, which is convenient for full-time staff to make weekly telephone return visits to understand the patient's emotions and life dynamics and give timely guidance and suggestions to help patients relieve stress and emotions. Regular quarterly communication seminars are held for discharged patients to provide a platform for communication, learning, and consultation. (4) Psychological regulation: on the one hand, by creating a warm and comfortable ward environment during hospitalization, such as placing green plants, the patient's psychology can be regulated. On the other hand, nursing staff should guide patients to carry out psychological exercises in a timely manner through verbal catharsis and deep breathing methods to help patients maintain a good psychological state, as shown in Figure 5.

Both groups were given intraperitoneal drugs such as hepatoprotective, antiviral, immunomodulatory, and enzyme-lowering and were hospitalized for observation for 2 weeks. Patients in the control group were given a routine model that included explaining that heparin is B-related knowledge, daily precautions (isolating saliva and blood-related items such as toothbrushes, towels, and razors from others), following medication recommendations, maintaining a positive therapeutic mindset, and paying attention to appropriate exercise, Aphrodite spicy diet, and overeating. Instruct the patient to review regularly at the time of discharge.

### 3.3. Evaluation Indicators

(1) The self-management scale (PIH, a means of assessing the psychological state of the meditators) was used to assess the management ability of two groups of patients, including self-monitoring, disease knowledge acquisition, and core management ability, with a total score of 88 points, and the higher the score, the poorer the management. (2) Before and after 1 month of nursing, the quality of life of two groups of patients was assessed using the Quality of Life Measurement Summary Table (QOL-BREF), including four dimensions of physical, psychological, social, and environmental fields, with a score of 100 points; the higher the score, the better the quality of life.

(1) $$\begin{array}{c} \text{SAS}=\text{Score}\times 1.25. \end{array}$$

Patients were followed up for 1 month after discharge and compared the treatment of the two groups. (1) The anxiety self-assessment scale (SAS) was used to evaluate the patient's anxiety level, and the depression self-assessment scale (SDS) was used to evaluate the patient's depression level, using SAS20 items, each with a score of 1 to 4 points, and the total score ×1.25 points: mild anxiety: 50-59 points; moderate anxiety: 60-69 points; severe anxiety: SAS ≥ 70 points; mild depression: 53-62 points; moderate depression: 63-72 points; and major depression: SDS ≥ 73 points. (2) Evaluation of patient treatment compliance: these 7 items include compliance with medication, not stopping medication without authorization, not eating and drinking, quitting smoking and alcohol, maintaining a good mental state, working and resting regularly, regularly reviewing, and those who are able to perform all of these tasks are considered fully compliant, those who cannot do any of the above are not compliant, and the rest are considered partially compliant. (3) The short life scale (SF-36) was used to evaluate the quality of life of patients. SF-36 includes 8 dimensions of general health (GH), bodily function (PF), bodily function (RP), somatic pain (BP), vitality (VT), social functioning (SF), emotional functioning (RE), and mental health (MH). Each dimension is rated from 0 to 100, and the higher the score, the better the quality of life.

(2) $$\begin{array}{c} \text{SF}=\overset{8}{\underset{i=1}{\sum }}c_{i}\cdot {\text{Score}}_{i}. \end{array}$$

### 3.4. Statistical Methods

In our research, we mainly use hypothesis tests for data processing, mainly including *t*-tests, *Z* tests, and chi-square tests. We consider the sample to conform to the normal distribution, i.e.,

(3) $$\begin{array}{c} x\sim N\left(\mu ,\sigma^{2}\right). \end{array}$$

First, establish the hypothesis of nothingness H0: *μ*1 = *μ*2; i.e., assume that there is no significant difference between the two population means. Then calculate the statistic *T*-value and use different statistical calculation methods for different types of problems. If you want to determine the degree of difference between the mean of a small sample in the population and the mean of the population, the formula used to calculate the *T*-value of the statistic is

(4) $$\begin{array}{c} T=\frac{\bar{X}-\mu_{0}}{s/\left(n-1\right)}. \end{array}$$

If you want to determine the degree of difference between the means of the two sets of samples, the *T*-value of the statistic is calculated as follows:

(5) $$\begin{array}{c} T=\frac{\bar{X_{1}}-\bar{X_{2}}}{\sqrt{\left(\sum x_{1}^{2}+\sum x_{2}^{2}\right)/\left(n_{1}+n_{2}-2\right)}\times \left(n_{1}+n_{2}\right)/\left(n_{1}\times n_{2}\right)}. \end{array}$$

The *Z* test is a commonly used method for large sample mean difference tests (that is, sample sizes greater than 30). It uses standard normal distribution theory to infer the probability of a difference occurring, thereby comparing whether the difference between the two means is significant.

(6) $$\begin{array}{c} Z=\frac{\bar{X}-\mu_{0}}{s/\sqrt{n}}, \end{array}$$

(7) $$\begin{array}{c} Z=\frac{\bar{X_{1}}-\bar{X_{2}}}{\sqrt{\left(s_{1}/n_{1}\right)+\left(s_{2}/n_{2}\right)}}. \end{array}$$

Chi-square testing is a hypothesis testing method used for various counting data. It falls under the category of nonparametric tests, which are primarily compared to two or more sample rates (composition ratios) and correlation analysis of two categorical variables. The basic idea is to compare the degree of coincidence or fitting between the theoretical frequency number and the actual frequency number.

(8) $$\begin{array}{c} \chi^{2}=\frac{\left(n-1\right)S^{2}}{\sigma^{2}}\sim \chi^{2}\left(n-1\right), \end{array}$$

(9) $$\begin{array}{c} \text{F}=\frac{S^{1}/S^{2}}{\sigma_{1}^{2}/\sigma_{2}^{2}}\sim F\left(n_{1}-1,n_{2}-1\right). \end{array}$$

To measure the final result, we test it with the probability *P* value of the sample observations or the more extreme result obtained when the null hypothesis is true; if the *P* value is small, the probability of the original hypothesis is very small; if it is true, then according to the principle of small probability, we have reason to reject the null hypothesis, and the smaller the *P* value, the more sufficient the reasons for our rejection of the null hypothesis. In summary, the smaller the *P* value, the more pronounced the results. However, whether the test result is “significant,” “moderately significant,” or “highly significant” needs to be solved according to the size of the *P* value and the actual problem.

(10) $$\begin{array}{c} p=\left\{\begin{array}{c} 2\left[1-\phi \left(Z_{0}\right)\right],\;p\neq p_{0},\\ 1-\phi \left(Z_{0}\right),\;p>p_{0},\\ \phi \left(Z_{0}\right),\;p<p_{0}. \end{array}\right. \end{array}$$

Use SPSS 23.0 statistics software to process data. The count data is expressed as *n* (%) ×^2^ and represented by the test. The measurement data is represented by the cloud $\bar{x}\pm$, using in-depth sample *t*-tests between groups and paired samples within groups. *P* < 0.05 indicates that the difference is statistically significant.

## 4. Results Analysis and Discussion

### 4.1. Management Capabilities

Before nursing, the PIH scores of the two groups were compared, and the difference was not statistically significant (*P* > 0.05). After one month of nursing, the PIH scores of both groups were lower than before nursing care, and the PIH scores of the observation group were significantly lower than those of the control group, and the difference was statistically significant (*P* < 0.05). See Table 1.

### 4.2. Quality of Life

QOL-BREF scores were compared between the two groups before nursing treatment, and the difference was not statistically significant (*P* > 0.05). After one month of treatment, the QOL-BREF scores of both groups improved compared with before treatment, and the QOL-BREF scores of the observation group were significantly higher than those of the control group, and the difference was statistically significant (*P* < 0.05). See Table 2.

### 4.3. Changes in SAS and SDS Scores before and after the Two Groups of Interventions

The SAS and SDS scores of the two groups were close before the intervention, and the difference was not statistically significant. After the intervention, the above scores in the observation group were lower than those in the control group, and the difference was statistically significant, as shown in Table 3.

### 4.4. Comparison of Treatment Adherence between the Two Groups

Treatment adherence was significantly better in the observation group than in the control group, with statistically significant differences (×^2^ = 10.85, *P* < 0.01), as shown in Table 4.

### 4.5. Changes in SF-36 Scores before and after the Two Groups of Interventions

The SF-36 scores of each dimension in the first two groups of the intervention were similar, and the difference was not statistically significant. After the intervention, the observed score was higher than that of the control group, and the difference was statistically significant, as shown in Table 5.

### 4.6. Analysis

Hepatitis is a chronic infectious disease that is difficult to treat. Studies have found that patient cognitive and management skills are a powerful way to prevent hepatitis. However, the existing basic methods can no longer meet the needs of hepatitis patients and their families. The nursing method can help patients recover by intervening in the cognition and life of patients with hepatitis and quickly and effectively improve the patient's management level and quality of life. The data of this scientific research shows that compared with the experimental group, after the observation group nursed 1 yuan, the management level PICH score was relatively low, the Clenlonzo score was relatively high, the difference was statistically significant, and the nursing mode used for patients with hepatitis could effectively quality their management level and life. According to the effective intervention of patients' rest, fitness time, and dietary structure, a warm ward environment is generated to ensure adequate sleep time and balanced nutritional intake of patients and to adjust anxiety. At the same time, effective communication is establishing a good doctor-patient relationship, so that nursing staff can deeply understand the dynamics of the patient's mentality, give immediate and accurate psychological counseling to the patient, and maintain the patient's attitude of close cooperation with the treatment. In addition, cognitive behavioral care interventions include knowledge education of patients' families, enabling them to achieve a united front between relatives and caregivers. The emotional care and suggestions of family members can effectively improve the patient's mentality, reduce anxiety, antitreatment, and other negative emotions, and maximize the efficacy under the premise of active treatment of patients.

It can be seen that improving health education knowledge in the clinical medical treatment of patients with diffuse hepatitis can improve the patient's ability to adapt to treatment, maintain a stable mentality, cooperate with each other in a variety of treatment and nursing, and improve their efficacy and quality of life. Many patients with diffuse hepatitis do not have enough knowledge of disease and treatment health education, which is easy to cause misunderstandings and cognitive dissonance, and cannot adequately cooperate with each other in treatment and care. Coupled with the influence of the patient's own bad living habits, the efficacy is weak. According to the specific situation of patients, targeted health guidance is carried out, and health education knowledge is optimized from multiple aspects such as patient mentality, diet structure, drug interaction, and lifestyle. Maximize the patient's treatment and nursing requirements, ensure a better concept of mutual cooperation between treatment and nursing, improve the trust of medical staff, and closely cooperate with various types of treatment and nursing to achieve overall efficacy.

This dissertation data showed that the SAS and SDS scores in the postintervention observation group were significantly lower than those in the control experiment, showing that the comprehensive nursing intervention could effectively improve the patient's negative mood and maintain optimism and positivity. The treatment compliance and SF-36 scores of the postintervention observation group were higher than those of the control group, indicating that the integrated nursing intervention could deepen the patient's understanding of the disease, build confidence in overcoming the disease, and improve treatment compliance and quality of life. Therefore, comprehensive nursing interventions can effectively alleviate the recovery of patients with hepatitis, the personal behavior of the doctor, and the quality of life.

## 5. Conclusion

Hepatitis B is a common infectious disease of the Chinese biliary system software. According to the type of disease, it can be divided into diffuse and subacute. Diffuse hepatitis is a multiple disease that seriously endangers the healthy life of patients. Clinical observation is based on antiviral therapy, which is difficult to treat and easy to attack. The greater the effectiveness, the less effective it is, creating a vicious circle. How to find efficacy, it is necessary to gradually improve the relevant treatment and care plan. According to the treatment compliance of the two groups after intervention, the treatment compliance rate of the intervention group was significantly higher than that of the control experiment 70.0%, and the difference was statistically significant (Ma Yili 0.05), which was consistent with the views reported by Li Fafang and others, and the treatment difficulty coefficient and long-term treatment of comprehensive nursing intervention hepatitis were lagging behind, which was easy to cause patients to have relatively large psychosomatic stress reactions, depression, anxiety, and other mental health problems. Reduce the patient's self-fire evacuation and confidence, lead to inconfidence and frustration in daily life such as diet and difference, and reduce the patient's self-efficacy. Therefore, patients must be given the necessary psychological guidance, which is conducive to self-efficacy.

Through the implementation of comprehensive nursing interventions, this scientific research makes the patients with hepatitis have obvious nursing ability, can quietly distribute daily life, and moderately change the living methods such as avoiding alcohol, taking medicine on time, regular physical examination, and maintaining a stable mentality. This study shows that the health education knowledge level, self-awareness, self-obligation, and self-care professional skills of patients in the post-ESCA scoring intervention group are higher than those in the preintervention group and the control experiment, and the difference is statistically significant, which is consistent with the reports of Ma Yili 0.05 and Li Zhuo, indicating that the self-reliance ability of comprehensive nursing intervention is beneficial to patients with hepatitis. Takizawa Ada's self-reliance ability is positively correlated with the patient's quality of life. The greater the ability to live on its own, the higher the quality of life. This study compared the scores of 2 groups of patients. The data showed that the physical disease and psychological and social development scores of the intervention group were significantly higher than those of the preintervention group and the control experiments, and the difference was statistically significant, which was consistent with the ten million miles view, reminding that the comprehensive nursing intervention was beneficial to the quality of life of patients with hepatitis. In general, based on comprehensive nursing interventions such as reasonable diet and medication consultation, maintaining a stable psychological state, and regular review for patients with hepatitis, patients' self-restraint ability and treatment compliance have been greatly improved. We conclude that the implementation of comprehensive nursing interventions is conducive to improving the treatment compliance and self-care ability of hepatitis B patients and improving their quality of life.

## Figures and Tables

**Figure 1:** Flowchart of hepatitis B prevention and treatment.

**Figure 2:** Functional role of the health system in the “five-party mode.”

**Figure 3:** Relationship between various factors in the management of patients with hepatitis B.

**Figure 4:** Clinical evolutionary pathways of hepatitis B.

**Figure 5:** Overall improvement in cognitive awareness of hepatitis B in patients in the test group.

**Table 1:** PICH scores ($\pm \bar{x}$, points) of self-management skills before and after nursing in two groups.

Constituencies	*n*	Before care	Postoperative care	*t*	*P*
Observation groups	71	66.55 ± 2.11	25.68 ± 4.32	71.629	0.001
Control group	71	66.23 ± 2.12	36.31 ± 3.55	60.972	0.001
*t*		0.902	16.019		
*P*		0.369	0.001		

**Table 2:** QOL-BREF scores before and after quality of life of patients in the two groups ($\bar{x}\pm$, score).

Constituencies	*n*	Before care	Postoperative care	*t*	*P*
Observation groups	71	71.65 ± 4.36	90.36 ± 5.48	22.513	0.001
Control group	71	71.71 ± 4.34	83.22 ± 5.41	13.984	0.001
*t*		0.082	7.813		
*P*		0.935	0.001		

**Table 3:** SAS and SDS scores before and after the two groups of interventions (scores, $\bar{x}\pm s$).

Constituencies	Number of examples	SAS		Safety data sheets	
		Before intervention	After intervention	Before intervention	After intervention
Control group	47	59.5 ± 9.7	51.3 ± 6.2	61.7 ± 10.6	54.9 ± 7.3
Observation groups	47	59.6 ± 9.8	36.8 ± 5.2	61.7 ± 10.5	39.8 ± 6.3
*t*，*P*		0.05, >0.05	12.29, <0.01	0, >0.05	10.74, <0.01

**Table 4:** Comparison of treatment adherence between the two groups (cases (%)).

Constituencies	Number of examples	Fully compliant	Partial compliance	B. noncompliance
Control group	47	18 (38.3)	15 (31.9)	14 (29.8)
Observation groups	47	29 (61.7)	16 (34.0)	2 (4.3)

**Table 5:** Changes in SF-36 scores before and after the two groups ($\bar{x}\pm s$).

SF-36 rating	Control group (*n* = 47)		Observation group (*n* = 47)	
	Before intervention	After intervention	Before intervention	After intervention
Somatotropin	62.1 ± 3.2	67.8 ± 6.6	61.4 ± 3.3	78.9 ± 5.6^∗^
Interrupter	63.1 ± 3.3	65.4 ± 5.2	62.8 ± 3.3	75.3 ± 5.2^∗^
RP	64.9 ± 2.8	67.7 ± 7.2	65.8 ± 2.6	77.1 ± 6.5^∗^
BP	64.8 ± 3.4	68.5 ± 6.3	65.3 ± 3.5	75.9 ± 5.4^∗^
Interrupter	65.9 ± 3.1	69.2 ± 6.7	66.5 ± 3.2	74.2 ± 7.2^∗^
SF	64.1 ± 4.2	67.4 ± 4.6	63.8 ± 4.2	72.3 ± 4.5^∗^
Again	62.1 ± 3.3	66.5 ± 5.3	61.2 ± 3.2	74.6 ± 5.5^∗^
Interrupter	61.8 ± 3.2	67.6 ± 6.6	62.3 ± 3.4	77.1 ± 5.4^∗^

^∗^Compared with the postintervention control group, *P* < 0.05.

## Data Availability

The labeled data set used to support the findings of this study is available from the corresponding author upon request.

## References

[1] Shrestha S., Tiwari P. S., Pradhan B. (2021). Occult hepatitis B infection in end-stage renal disease patients starting maintenance hemodialysis at a tertiary care hospital: a descriptive cross-sectional study. *Journal of Nepal Medical Association*.

[2] Younus I., Ali M. Z., Ajmal M., Akhtar H., Ali J., Altaf F. (2021). Burden and baseline characteristics of patients with decompensated liver disease in Tertiary Care Hospital Gujrat. *The Professional Medical Journal*.

[3] Asad M., Hameed S., Subhan M. (2020). Frequency of hepatitis B and C and their demographic status in voluntary blood donors in a tertiary care hospital. *AATM 2015*.

[4] Butt N., Hussain R., Rai L. (2020). Efcacy of pegylated interferon-alpha-2a in hepatitis D infected patients. *Experience from the Tertiary Care Hospital in Karachi.*.

[5] Khullar S., Parihar R. S., Khatri P. K. (2020). Seroprevalence of hepatitis B virus and hepatitis C virus infection in haemodialysis patients at tertiary care hospital in Western Rajasthan, India. *Journal of The Academy of Clinical Microbiologists*.

[6] Balasundaram P., Tiwari V. K., Raj T. S. (2020). Cost of treatment and consequences for chronic hepatitis B and C virus infection at a tertiary care hospital in Delhi. *Indian Journal of Public Health*.

[7] Omar N. (2021). Seropositivity of hepatitis B & C in hemodialysis patients at two tertiary care centers in Lahore. *BioMedica*.

[8] Deo R. K., Chitalkar P., Malla S., Kc I., Karki B., Thapa R. (2021). Epidemiology, clinico-radiological profile and management of hepatocellular carcinoma in a tertiary care venter in Nepal. *Medical Journal of Shree Birendra Hospital*.

[9] Shrestha S., Mahatara S., Pun S. B., Shrestha M., Napit R., Manandhar K. D. (2020). Serological markers and molecular analysis of hepatitis B infection in a tertiary care hospital at Kathmandu, Nepal. *Indian Journal of Gastroenterology*.

[10] Siakavellas S., Goulis J., Manolakopoulos S. (2020). Monitoring and comorbidities in patients with chronic hepatitis B currently treated with nucleos(t)ide analogs. *Annals of Gastroenterology*.

[11] Alshehail B., Alotaibi N., Joseph R., Alshayban D. (2021). A quasi-experimental trial of the clinical and economic impact of implementing of hepatitis B immunoglobulin policy post needle stick and sharp injuries in reducing its unnecessary use at a tertiary care hospital. *International Journal of Clinical Practice*.

[12] Durga B. (2021). Knowledge and preventive practices of hepatitis B transmission among dental students and interns in a tertiary hospital: a descriptive cross-sectional study. *JNMA; Journal of the Nepal Medical Association*.

[13] Nn A., Sf B. (2020). Seroprevalence of hepatitis B, hepatitis C and HIV 1/2 in patients undergoing surgery in a tertiary care hospital in north India (a hospital based study). *Clinical Epidemiology and Global Health*.

[14] Chhina D., Garg S., Chinna R., Dhiman P., Gupta D. (2020). Study of prevalence of hepatitis B, hepatitis C, and other opportunistic coinfections in HIV-infected patients in a tertiary care hospital of North India. *JOURNAL OF GASTROINTESTINAL INFECTIONS*.

[15] Sharma A., Najmeen S., Rauf A. (2020). Seroprevalence of hepatitis B surface antigen (HBSAg) among patients attending tertiary care teaching hospital in Solapur. *Maharashtra*.

[16] Sievert K., Liddle R., Tan A., Arachchi N., Valaydon Z., Allard N. (2020). Promoting hospital and primary care collaboration for timely and effective care for chronic hepatitis B in western Melbourne. *Australian health review: a publication of the Australian Hospital Association*.

[17] Gulalai N. A., Wahid A., Khan A., Atif M., Khan A. (2020). Evaluation of management and factors associated with hypertension control in hemodialysis patients at a tertiary-care hospital in Pakistan. *Perspectives*.

[18] Reid P., Kandasamy V., Chambers B. (2021). The benefits of a virtual ward model in the management of care of elderly patients admitted with decompensated heart failure. *Age and Ageing*.

[19] Gaikwad R. A., Gadappa S. N. (2021). Intrauterine balloon tamponade in the management of atonic postpartum haemorrhage: case study from a tertiary care hospital. *The New Indian Journal of OBGYN*.

[20] Ali S., Ahmed Z., Metlo M. (2021). Comparative study of compliance between sofosbuvir and interferon in the management of viral hepatitis at tertiary care hospital of Gambat, Sindh, Pakistan. *Journal of Pharmaceutical Research International*.

